# The Generation of Piano Music Using Deep Learning Aided by Robotic Technology

**DOI:** 10.1155/2022/8336616

**Published:** 2022-10-10

**Authors:** Jian Pan, Shaode Yu, Zi Zhang, Zhen Hu, Mingliang Wei

**Affiliations:** ^1^College of Music and Dance, Sichuan Film and Television University, Chengdu 611331, Sichuan, China; ^2^School of Information and Communication Engineeringn, Communication University of China, Beijing 100024, China; ^3^Information and Communication Engineeringn, Chengdu Medical College, Chengdu 610500, Sichuan, China; ^4^Science and Technology Training School of Qimengweilai, Chengdu 611000, Sichuan, China

## Abstract

In order to improve the accuracy and precision of music generation assisted by robotics, this study analyzes the application of deep learning in piano music generation. Firstly, based on the basic concepts of robotics and deep learning, the advantages of long short-term memory (LSTM) networks are introduced and applied to the piano music generation. Meanwhile, based on LSTM, dropout coefficients are used for optimization. Secondly, various parameters of the algorithm are determined, including the effects of the number of iterations and neurons in the hidden layer on the effect of piano music generation. Finally, the generated music sequence spectrograms are analyzed to illustrate the accuracy and rationality of the algorithm. The spectrograms are compared with the music sequence spectrograms generated by the traditional restricted Boltzmann machine (RBM) music generation algorithm. The results show that (1) when the dropout coefficient value is 0.7, the function converges faster, and the experimental results are better; (2) when the number of iterations is 6000, the error between the generated music sequence and the original music is the smallest; (3) the number of hidden layers of the network is set to 4. When the number of neurons in each hidden layer is set to 1024, the training result of the network is optimal; (4) compared with the traditional RBM piano music generation algorithm, the LSTM-based algorithm and the sampling frequency distribution tend to be consistent with the original sample. The results show that the network has good performance in music generation and can provide a certain reference for automatic music generation.

## 1. Introduction

In recent years, with the continuous development of theory and technology in the field of artificial intelligence (AI), its related research results have been widely used. For example, language recognition, image recognition, natural language processing, and other related achievements have brought a lot of convenience to all aspects of people's lives [1–4]. Robotics is one of the main technologies in the field of AI. Music robotics is a top-level applied discipline at the intersection of music and technology. Since the 21st century, music robot technology has been widely developed, including different technologies such as the principle of music robot pronunciation, expressive performance, bionic structure, and intelligence. As one of the symbols of “AI,” the problem of music generation by music robots has become a research hotspot [5]. The most important thing in the field of music style recognition and generation is the extraction of relevant features and the selection of classifiers. Different music feature vectors are selected for music style recognition, and different classification effects will be produced. At present, the identification of musical styles still uses features such as pitch, timbre, and loudness. If this study only relies on manually extracted features, the speed and accuracy of classification will be greatly reduced. In order to obtain a more accurate recognition effect, it is also necessary to deeply mine the intrinsic correlation between the data [6].

With the deepening of research, deep learning models have been widely used in music generation. These deep models include recurrent neural network (RNN), generative adversarial network (GAN), restricted Boltzmann machine (RBM), convolutional neural network (CNN), and long short-term memory (LSTM) [7]. In addition, the mixed-use of networks in reinforcement learning (RL) and deep learning is also used in music generation. Each algorithm has certain drawbacks. For RNN, since the network does not have the effect of long-term memory, the effect of the generated music is not very good. For GAN, the network is not very good at dealing with variable content. A problem that is easy to arise is adding some rhythms to the generated music that are different from the original music. RBMs are slightly insufficient in controllability. Some scholars have used the forward feature selection algorithm to extract the underlying features of music. These features include spectral center value, linear prediction coefficient, zero-crossing rate, and more than ten musical features. Music features are combined with multimodal analysis and identification methods to finally achieve the effect of music genre classification. It mainly contains five music genres: classical, country, pop, jazz, and rock. In addition, some scholars also perform music recognition by extracting the rhythm and pitch from the music features to form a two-dimensional feature vector and finally achieve the effect of music recognition [5, 8–11]. Hizlisoys et al. proposed a method for music emotion recognition based on a deep neural network (DNN) architecture with convolutional LSTM. The CNN layer provides log Mel filter bank energy and Mel frequency cepstral coefficients to obtain features. The classification results show that the best performance can be obtained when the new feature set is combined with standard features using LSTM fusion DNN classifiers [12]. Li et al. transferred DNN models to music classification and used spectrograms to evaluate the performance of the models, as shown by extensive experimental evaluations on three music datasets. The balanced trust loss function model, Resnet50_trust, consistently outperforms other DNN models [13].

Music genre identification and classification have been deeply analyzed in music robotics research. Deep learning is also used to generate music and has a certain research basis. As a very important part of deep learning, RNN has also made great strides in music generation. The network is very powerful in dealing with long-time series problems. However, using an RNN model only for simple music is not ideal. This paper introduces the related technologies and theories that are needed for different genres of music generation in deep learning and summarizes some key technologies currently used in music feature extraction. Based on the LSTM network, the music style recognition and generation networks are redesigned. The dimensions of the input network matrix and output matrix are designed to make training easier. The comparison between different spectrograms illustrates the accuracy of the experiment, and genre classification predictions are also performed on the generated music to illustrate that the network can generate music of different genres.

## 2. Introduction of Related Algorithms and Model Establishment and Training

### 2.1. Music Generation and Robots

As a creative artistic expression, music is the unique crystallization of human wisdom and emotion. Therefore, automatically generating music with a clear style and in line with the aesthetics of listening, especially different from existing music, has become one of the criteria for AI evaluation. This is also a hot spot for deep learning applications [14].

Most methods use the musical instrument digital interface (MIDI) as the notation of music [15]. Its advantages are that it is straightforward, the result of the model is the musical score, and the training data are easy to obtain. Its downside is the lack of support for intervals or chords. In addition, data augmentation of the song are required. The MIDI file contains only one way of playing a melody for the model to learn all the possibilities of this melody in the entire note definition domain. This not only requires the network to have higher capacity but also exacerbates the consumption of training resources.

At present, most of the research focuses on the performance of musical robots. Therefore, music generation is the “performance basis” of music robots. The intelligent generation of music by the music robot will improve the service level of the music robot. Music robots recognize more beats and styles, including some music style recognition and prediction systems based on spectrum information and feature extraction of the support vector machine (SVM) algorithm. In the past, most of the effort was devoted to featuring extraction. The quality of the features largely determines the result of classification and recognition. Although many features have been extracted to solve audio problems, direct features related to the structure are always difficult to describe. Today, the renewed development in the field of deep learning has made neural networks widely used in the field of audio processing. Therefore, this study uses deep learning technology to study the intelligent music generation of robots and strives to lay a certain foundation for the development of music robots.

### 2.2. Advantages and Features of MIDI

Although the MIDI format has many shortcomings in terms of neural network data set acquisition and data modeling, this study prefers symbol sequences that can accurately express information such as rhythm, timing, pitch, and velocity, rather than audio signals. Therefore, MIDI files are a more suitable choice as the input dataset for the network.

The standard midi format (SMF) of the standard MIDI format is composed of a series of chunk data blocks. Its header data block is a file, and immediately after the file header block is a track block that stores track information [16]. The parts included in the standard MIDI format file are shown in Figure 1.

### 2.3. Concepts Related to Deep Learning

Deep learning has further improved based on machine learning. Since the deep learning architecture contains more layers of networks, more features can be obtained when analyzing features. This can improve the learning ability of the network. Compared with shallow networks, deep networks can use fewer neurons to perform the same function and be more efficient and accurate in the learning process. Deep learning has been used in various fields, such as finance, security, and manufacturing [17].

#### 2.3.1. Neurons

Neurons are also called perceptrons. It is the most basic unit of neural networks. The neural network structure is shown in Figure 2.

In Figure 2, a complete neural network consists of an input layer, a hidden layer, and an output layer. The input layer is mainly used for input vectors. The hidden layer is used for vector analysis and parameter learning. The output layer is the output result. If the neural network has many hidden layers, it belongs to the category of deep learning [18]. Deep learning is mainly to study different DNNs, and then use DNNs to solve different problems.

The perceptron algorithm solves a lot of problems. The composition of a perceptron is shown in Figure 3.

The initial value of the weight W of the perceptron model is generally set randomly, which often fails to achieve a good fitting result. Therefore, it is necessary to calculate the output value and then make the difference between the actual output value and the theoretical output value to adjust each output. The learning rule is an algorithm used to calculate a new weight matrix W and a new bias *b*. The input layer input is a vector (*m*_1_, *m*_2_, *m*_3_, ⋯, *m*_*n*_丨*m*_*i*_ ∈ *R*). Each input corresponds to a weight *w*. Additionally, the other bias is *b*. The value of the offset is generally 1, denoted as *w*_0_. The sum of weight values is calculated as shown in the following:

(1) $$\begin{array}{c} z=\overset{n}{\underset{i=1}{\sum }}w_{i}m_{i}+b\text{.} \end{array}$$

The output value can be denoted as *y*. The value of *y* can be calculated by the activation function *g*(*z*). There are many choices of activation functions, as shown in the following:

(2) $$\begin{array}{c} y=g\left(x\right)\text{.} \end{array}$$

#### 2.3.2. Feedforward Neural Network

Multiple neurons are interconnected to form a neural network. The feedforward neural network (FNN), composed of a single layer of neurons, is shown in Figure 4.

In Figure 4, the single-layer neuron feedforward network has four input units and three neurons as output units. Each input unit feeds forward to the output layer of each neuron. This two-layer neuron structure is also called a perceptron. Another common network structure is a multilayer FNN. Its basic structure is like a single-layer feedforward network, but there are some additional hidden layers between the input and output layers. Neural networks can extract higher-order and global data based on these hidden layers. Neural network knowledge is acquired through the network's learning process on the dataset. Among them, the weights of the synapses are continuously adjusted in order to match the network output with the desired output. This approach is also known as supervised learning. The learning ability of multilayer networks is much stronger than that of single-layer perceptrons. Among them, the most commonly used method for training multilayer networks is the backpropagation algorithm. It is the most successful neural network learning algorithm and can be used not only for multilayer FNN but also for other networks, such as RNN. The algorithm is based on the gradient descent strategy, and the difference between the expected value of the network and the actual output is sent back to the input, so the current learning situation of the network can be obtained. Usually, a loss function is used to express this criterion [19–21].

The most used loss function is the mean squared error. For the training data sample (*x*^*n*^, *t*^*n*^), assuming that the output of the neural network is ${\bar{t}}^{\left(n\right)}$, the mean square error of the neural network on this sample is calculated as shown in the following:

(3) $$\begin{array}{c} E_{n}=\frac{1}{2}\overset{l}{\underset{j=1}{\sum }}{\left({\bar{t}}_{j}^{n}-t_{j}^{n}\right)}^{2}\text{.} \end{array}$$

#### 2.3.3. Gradient Descent

The gradient descent algorithm is relatively efficient. By using this algorithm, it is relatively easy to obtain the optimal solution for the function that needs to be trained, thereby improving the accuracy of the model. The method can be divided into three categories, namely batch gradient descent, mini-batch gradient descent, and stochastic gradient descent [22].

When this function is derivable, by calculating the inverse of the function, the optimal solution *θ* of the training function is regarded as a variable, and the optimal solution can be obtained. Additionally, the calculation of the weights also needs to be adjusted according to the learning rate *η*. The update of *θ* is shown in the following:

(4) $$\begin{array}{c} \theta =\theta -\eta \nabla_{\theta }J\left(\theta \right). \end{array}$$

In the actual application process, the update of *θ* takes a long time. Therefore, in the process of training with large batches of data, it is difficult to complete the training online. For larger datasets, the training process may be harder because more memory is required.

One disadvantage of the stochastic gradient descent algorithm (SGDA) is that it is only suitable for training datasets. Each set of training data can calculate the gradient. For example, there is a set of training data (*x*^*i*^; *y*^*i*^), the value of *i* belongs to (0, *n*), and *n* represents the size of the entire data set. The update of *θ* is shown in the following:

(5) $$\begin{array}{c} \theta =\theta -\eta \nabla_{\theta }J\left(\theta ;x^{i};y^{i}\right)\text{.} \end{array}$$

Since this method is aimed at the training dataset, and only one sample is randomly selected to update the parameters at a time, the learning efficiency of this method is very high, and it can be updated online. The only downside is that there will be optimization fluctuations due to updates not going in the right direction. In general, the advantages of SGDA are still obvious, and it is relatively easy to find better local minimum points.

The mini-batch gradient descent algorithm is derived from the two algorithms mentioned above. The algorithm needs to find a balance point in the process of updating, and each update will select fewer samples than *n* from the training set. *θ* is updated as shown in the following:

(6) $$\begin{array}{c} \theta =\theta -\eta \nabla_{\theta }J\left(\theta ;x^{\left(i:i+n\right)};y^{\left(i:i+n\right)}\right)\text{.} \end{array}$$

Compared with the batch gradient descent algorithm, the mini-batch gradient descent algorithm greatly improves the learning efficiency of the mini-batch algorithm. It does not require a large amount of memory. It is also more efficient when performing matrix operations. Therefore, the mini-batch gradient algorithm is one of the most used algorithms in neural networks.

#### 2.3.4. LSTM

LSTM is a special type of RNN. Its purpose is to solve the long-term dependency problem of traditional RNN. It is designed to avoid the rapid decay of back-propagated errors [23]. The storage unit structure of the LSTM network is shown in Figure 5.

In Figure 5, a single storage unit in a conventional RNN neuron is replaced with a storage block containing multiple storage units. They can pass memory cell values down multiple time steps along the time axis and can be memorized or forgotten at each time beat. It can capture the information and dependencies of long-distance steps, which is a very necessary function for the extraction of abstract musical features. Therefore, it is a more appropriate choice for the LSTM network to be applied to the generation of musical melodies [24].

The current state of a memory cell depends on its previous state, the network itself, the forget gate, and the input value of the input gate. The neuron state update is shown in the following:

(7) $$\begin{array}{c} S_{c}=S_{c}y^{\varphi }+g\left({net}_{c}\right)y^{in}\text{.} \end{array}$$

After the input vector enters the neuron, through the activation function, *g*() squeezes the input value into the interval of 0 to 1 and then multiplies the input value obtained by the input gate. The process is shown in the following:

(8) $$\begin{array}{c} y^{in}=\sigma \left({net}_{in}\right)\text{.} \end{array}$$

Among them, *σ*() represents the sigmoid activation function. When *y*^in^ is 0, by multiplying *g*(net_*c*_) and *y*^in^, the input gate can prevent the network input net_in_ from updating the neuron storage unit.

Like in the calculation process of *y*^in^, the output value *y*^*c*^ of the neuron is the storage unit state *s*_*c*_. After being squeezed through the activation function *h*(), it is multiplied by the value *y*^out^ of the output gate, as shown in the following:

(9) $$\begin{array}{c} y^{out}=\sigma \left({net}_{out}\right)\text{,} \end{array}$$

(10) $$\begin{array}{c} y^{c}=h\left(s_{c}\right)y^{out}\text{.} \end{array}$$

### 2.4. Implementation and Training of a Music Generation Model Based on Deep Learning

#### 2.4.1. Training and Testing Data

The MIDI music website selects relevant data (musescore.com) and selects ten genres. One hundred music clips are selected for each music genre, for a total of 1000 music clips. The time of each song is different, generally between the 30 s and 300 s. All data are in MIDI music format. In the experiment, five groups of music were selected for analysis. The number of training and test sets for all groups is 180 and 20, respectively. The amount of data per genre is 200.

#### 2.4.2. Network Training and Optimization

The neural network uses Python 3.10.6 to write the entire system, uses Tensorflow to implement the programming language framework, and uses Music21 for music classification. Training of the network: after all model parameters are determined, the network is trained. In the training process, the training data are used, and the updated parameters are selected repeatedly to optimize the model performance [25]. During the training process, the values of some hyperparameters in the model are set, such as the number of iterations and the number of network layers and hidden layer units.  Figure 6 shows the training process of the music generation algorithm.

In Figure 6, after the network is trained, it can generate music of different genres. The music generation network generates a new note, mainly by combining the previous input note with the current input note and then making predictions [26]. Here, all notes are converted into vectors, which are used to compare and predict. The detailed flow chart of music sequence generation is shown in Figure 7.

In Figure 7, first, the trained network and the set parameters are loaded. N represents the length of the sequence. If the sequence length is greater than 0, forward propagation is performed, and the value of the loss function is calculated. Here, there is a threshold. If the value of the loss function is already smaller than the threshold, it means that the music feature vector is valid at this moment, and the next moment's sequence value is predicted. Finally, the entire sequence of predicted music is output.

*(1) Network Optimization*. During training, when the dataset is small, a common problem is overfitting. The generalization ability is poor, and the consequence is that the effect of the model is not good and the accuracy is not enough. In order to prevent the overfitting problem and improve the accuracy of the network, the experiment adopts the dropout method. A dropout refers to randomly ignoring the weights of some hidden layer nodes when training a neural network [27]. During training, these nodes will not work. Their weights are also not updated. Dropout is added between hidden layers, as shown in the following:

(11) $$\begin{array}{c} r=\left(1-p\right)xf\left(W_{v}+b\right)\text{.} \end{array}$$

Here 1 − *p* is a binary model that follows the Bernoulli distribution. When the probability value is *p*, the value is 1, and the rest is 0. In the experiment, all parameters are multiplied by *p* to achieve the purpose of changing the parameters [28, 29].

## 3. Experimental Results

### 3.1. Network Optimization Results

In this experiment, in order to optimize the performance of the model, the convergence effect of the loss function in the three cases of *p*=0.5, *p*=0.6, and *p*=0.7 is analyzed separately. The convergence effect of the loss function is shown in Figure 8.

In Figure 8, when the probability value is *p*=0.5, the convergence value is 0.0035, which is larger than when *p*=0.7. At *p*=0.6, the experimental effect is better than at *p*=0.5 but not as good as at *p*=0.7. Therefore, the experimental results are best when the probability value is *p*=0.7. Finally, the dropout coefficient value of this model is determined to be 0.7.

### 3.2. Analysis of Algorithm Influencing Factors

According to the experience of neural network training and as the number of iterations of the LSTM network increases, the experimental error will become smaller and smaller [30–32]. The data means that the closer the actual output value is to the target value, the closer the training result is to the target value, as shown in Figure 9.

In Figures 9(a) and 9(b), after 3000 iterations, the frequency distribution of the generated music sequence is roughly the same as the original music sequence frequency distribution, but there are still some obvious differences. For example, the generated music sequence spectrogram contains many frequencies, not in the original music sequence spectrum. In Figure 9(c), after 6000 iterations, the generated music spectrogram is completely consistent with the original music spectrogram. The main reason is that with the increase in the number of iterations, the model parameters are also updated many times. Finally, the parameters of the model are optimized.

The effect of the number of neurons in the hidden layer of the neural network on the experiment is analyzed. The influence of the hidden layer neurons on the experimental error is shown in Figure 10.

In Figure 10, when the number of neurons in each layer is 128, 256, 512, and 1024, in turn, the training results become more and more accurate, and the error value becomes smaller and smaller. If the number of neurons is too large, the computer environment is very demanding, and the training time will increase geometrically, increasing the complexity by several degrees. Therefore, the number of neurons in the network's hidden layer is 1024, which can make the training result optimal.

During the experiment, the spectrum analysis is performed on the music sequences generated by the model under different hidden layers in turn. The generated music spectrograms and sample spectrograms are shown in Figure 11.

In Figure 11, the effect of LSTM on music analysis is still obvious. With the increased number of neural network layers, the trained music spectrogram is getting closer and closer to the original spectrogram, indicating that its accuracy is getting higher and higher. When there are two hidden layers, some frequencies do not appear. When the hidden layer has four layers, the difference between the generated music sequence and the original music sequence is very small, which shows that the generated music is the most accurate when there are four hidden layers.

The LSTM-based music generation algorithm is compared with the traditional RBM music generation algorithm, and the spectrograms of the music generated by the two generative models are analyzed separately. The results of the music spectrogram generated by the two methods are shown in Figure 12.

In Figure 12, the trend of the spectrograms of the music generated by the traditional RBM and the original music is highly similar. However, RBM-generated music is not as accurate as LSTM-generated music. In Figure 12(a), when the frequency of the original sample music is around 1000–2000 Hz, the voltage value exceeds 35, and Figure 12(b) does not exceed. Compared with Figure 12(c), the music spectrogram generated by LSTM is more consistent with the original music spectrogram in both the overall frequency distribution and the sample frequency distribution.

## 4. Conclusion

This experiment mainly analyzes the experimental effect of deep learning in piano music generation under robotics technology. The music sequence spectrograms are analyzed to illustrate the accuracy and rationality of the algorithm. Firstly, based on introducing the basic concepts of deep learning, the advantages of the LSTM network in music generation are introduced. Meanwhile, dropout coefficients are used to optimize the neural network. Through experimental verification, the dropout coefficient value is 0.7. Secondly, this experiment analyzes the experimental effect of the algorithm, including the influence of the number of iterations and neurons in the hidden layer, on the effect of music generation. When the number of iterations is 6000, the error between the generated music sequence and the original music is the smallest. When the number of hidden layers of the network is set to 4 and the number of neurons in the hidden layer is set to 1024, the training results of the network are best. Spectrograms of sequences generated by music generation algorithms based on LSTM and traditional RBM show that neural networks perform well in music generation. The shortcomings of this study that can be improved in the future are (1) due to limited energy, the music training dataset selected is small, and the music styles are similar. The internal structure and logic of different styles of music are not similar. If it is mixed together to generate music, the accuracy will be much less. Future research will focus on how the more complex data can be separated from other multitrack data. The processing of the data of these tracks enables the neural network to process and analyze the multitrack data. (2) This experiment mainly extracts digital features of music, including pitch, timbre, and loudness. Other features can be extracted later, such as energy features and time domain features. Rich data features lead to better results. (3) The algorithm model finally generates a matrix containing music features, which also needs to be converted into playable music. Future research could be considered to include how to automatically generate music without the need to reverse the process.

## Figures and Tables

**Figure 1:** Standard MIDI format file.

**Figure 2:** The structure diagram of the neural network.

**Figure 3:** Perceptron diagram.

**Figure 4:** The network of single-layer neuron feedforward.

**Figure 5:** Storage unit structure of LSTM network.

**Figure 6:** Flow chart of music generation training.

**Figure 7:** Flow chart of music sequence generation.

**Figure 8:** Function convergence diagram under different *p* values.

**Figure 9:** Music spectrogram under different iterations. (a): Spectrogram of original sample music sequence; (b): spectrogram of music sequence iterated 3000 times; and (c): Ssectrogram of music sequence iterated 6000 times.

**Figure 10:** The effect of the number of neurons in the hidden layer on the error.

**Figure 11:** Spectrogram of music with different hidden layers. (a): Spectrogram of sample music sequence; (b): spectrogram of music when the hidden layer is 2; and (c): spectrogram of music when the hidden layer is 4.

**Figure 12:** Music spectrograms of the two algorithms. (a): Original music spectrogram; (b): RBM-generated music spectrogram; and (c): LSTM-generated music spectrogram.

## Data Availability

The raw data supporting the conclusions of this article will be made available by the authors, without undue reservation.
